# Overexpression of α-synuclein in oligodendrocytes does not increase susceptibility to focal striatal excitotoxicity

**DOI:** 10.1186/s12868-015-0227-6

**Published:** 2015-12-02

**Authors:** Daniela Kuzdas-Wood, Lisa Fellner, Melanie Premstaller, Carlijn Borm, Bastiaan Bloem, Deniz Kirik, Gregor K. Wenning, Nadia Stefanova

**Affiliations:** Division of Neurobiology, Department of Neurology, Medical University of Innsbruck, Innrain 66/G2, 6020 Innsbruck, Austria; Department of Neurology, Parkinson Center Nijmegen (ParC), Radboud University Nijmegen Medical Centre, Nijmegen, The Netherlands; Department of Experimental Medical Science, BMC D11, Brain Repair and Imaging in Neural Systems (BRAINS), Lund University, Klinikgatan 32, 22184 Lund, Sweden

**Keywords:** Excitotoxicity, Alpha-synuclein, Quinolinic acid, Neurodegeneration, Striatum, Multiple system atrophy

## Abstract

**Background:**

Multiple system atrophy (MSA) is a fatal adult-onset neurodegenerative disease characterized by α-synuclein (α-syn) positive oligodendroglial cytoplasmic inclusions. The latter are associated with a neuronal multisystem neurodegeneration targeting central autonomic, olivopontocerebellar and striatonigral pathways, however the underlying mechanisms of neuronal cell death are poorly understood. Previous experiments have shown that oligodendroglial α-syn pathology increases the susceptibility to mitochondrial stress and proteasomal dysfunction leading to enhanced MSA-like neurodegeneration. Here we analyzed whether oligodendroglial α-syn overexpression in a transgenic mouse model of MSA synergistically interacts with focal neuronal excitotoxic damage generated by a striatal injection of quinolinic acid (QA) to affect the degree of striatal neuronal loss.

**Results:**

QA injury led to comparable striatal neuronal loss and optical density of astro- and microgliosis in the striatum of transgenic and control mice. Respectively, no differences were identified in drug-induced rotation behavior or open field behavior between the groups.

**Conclusions:**

The failure of oligodendroglial α-syn pathology to exacerbate striatal neuronal loss resulting from QA excitotoxicity contrasts with enhanced striatal neurodegeneration due to oxidative or proteolytic stress, suggesting that enhanced vulnerability to excitotoxicity does not occur in oligodendroglial α-synucleinopathy like MSA.

## Background

Multiple system atrophy (MSA) is an adult-onset, progressive, neurodegenerative disorder with unknown etiology. MSA presents with levodopa-resistant Parkinsonism, cerebellar ataxia, pyramidal signs and autonomic failure in any combination [1]. The main pathological hallmark of MSA is the occurrence of α-synuclein (α-syn)-positive glial cytoplasmic inclusions (GCIs) that are predominantly found in oligodendroglial cells [2]. MSA is thought to be a primary oligodendrogliopathy [3]. Furthermore, striatonigral degeneration (SND) and olivopontocerebellar atrophy (OPCA) are described to underlie the motor symptoms [4, 5]. Although the occurrence of GCIs is recognized as a fundamental factor in the pathogenesis of MSA, the association of GCIs with neuronal degeneration in MSA remains unclear. In addition, neuroinflammation, excitotoxicity, proteasomal dysfunction and oxidative stress are thought to be involved in the neurodegenerative process of MSA [6–11]. Experimental models provide an important tool to study the disease mechanisms and test new therapeutic targets in MSA [12]. The development of a transgenic mouse model which reproduces GCI-like aggregations by overexpression of α-syn under control of the proteolipid-protein promoter (PLP) [13] or the myelin basic protein (MBP) [14] in oligodendroglial cells has been instrumental to address mechanisms of MSA-like neurodegeneration [12, 15–19]. Systemic exposure of transgenic PLP-α-syn mice to the mitochondrial toxin 3-nitropropionic acid (3-NP) resulted in dose-dependent MSA-like neurodegeneration supporting the role of systemic oxidative stress in the pathogenesis of this disorder [12, 20]. Oligodendroglial α-syn overexpression in PLP-α-syn mice as well as MBP-α-syn mice resulted in increased 3-NP vulnerability associated with oxidative changes of α-syn pathology in oligodendrocytes that may partly mediate the enhanced neuronal vulnerability to systemic stress [12, 21, 22]. Supporting this notion, systemic exposure to proteasome inhibition triggered wide-spread MSA-like neurodegeneration in transgenic PLP-α-syn mice but not in wild type controls highlighting the importance of aggravated oligodendroglial α-syn pathology through systemic proteolytic stress for increased neuronal vulnerability [23].

Abnormally enhanced glutamatergic neurotransmission may cause excitotoxic cell damage and lead to neuronal death that has been classically associated with Huntington’s disease [24] and amyotrophic lateral sclerosis [25] among others. Excitotoxic neuronal injury has been suggested in MSA [10] but the evidence is sparse. Alternatively, a large phase III randomized placebo-controlled trial of riluzole, an anti-excitotoxicity drug, failed to modify overall severity and progression in MSA [26] adding to the controversy on the role of excitotoxicity in this disorder.

Quinolinic acid (QA) is a useful tool to address excitotoxic pathways in models of neurodegenerative disorders. QA is known for its potential to selectively activate the *N*-methyl-d-aspartate (NMDA) sensitive subpopulation of glutamate receptors [27]. It has been shown that already minimal amounts of QA can directly activate NMDA receptors or lead to the release of endogenous glutamate and thus induce significant neuronal damage [28, 29]. In the present work we aimed to combine stereotactic striatal QA lesions with the oligodendroglial α-syn pathology in the transgenic PLP-α-syn MSA mouse model to identify whether the preceding α-syn toxicity may enhance excitotoxic injury and striatal neuronal loss and thus play a specific role in MSA pathogenesis. Therefore, QA was stereotactically injected into the striatum of transgenic PLP-α-syn and control mice. The excitotoxin-induced motor impairment and striatal neuronal loss was comparable in transgenic PLP-α-syn and control mice.

## Methods

### Animals and surgery

This animal experiment was performed in accordance with the ethical guidelines and with the specific permission of the Ethics Committee at the Austrian Federal Ministry of Science and Research (BMWF-66.011/0041-II/3b/2011). All efforts were made to minimize animal suffering and to reduce the number of animals used. The mice were housed under 12 h light/dark-cycle with free access to food and water. In the present study we used seven-month old transgenic PLP-α-syn mice (n = 8) and age-, sex- and background-matched healthy control mice (n = 7). To assess the effects of QA all animals received stereotaxic injections of 90 nmol QA (Sigma-Aldrich, USA) into the left striatum (AP +0.7 mm, ML +2.0 mm, V −3.0 mm) under deep inhalation isoflurane (Abbott, USA) anaesthesia using 4 vol % for induction and 1.5–2 vol % intrasurgically.

### Behavioral tests

Behavioral tests were done 15 weeks post surgically to assess the effects of QA striatal lesion.

#### Open field activity

To investigate the locomotor activity of the two groups the flex field activity test (San Diego Instruments, USA) was performed as previously described [12]. Briefly, mice were placed in the center of the open field (40.5 × 40.5 × 36.5 cm) and the horizontal and vertical (rearing) locomotor activity was measured for 15 min. The tests were performed in a dark room with complete isolation from external noises during the test period.

#### Drug induced rotations

The well-established automated rotometer system (San Diego Instruments, USA) was applied to assess rotational asymmetry as described previously [30, 31]. Amphetamine-induced rotations were measured for 60 min upon intraperitoneal injection of d-amphetamine sulfate (5 mg/kg, dissolved in 0.9 % sterile saline, Sigma-Aldrich, Austria). Apomorphine-induced turnings were quantified for 60 min upon subcutaneous apomorphine hydrochloride injections (0.5 mg/kg, dissolved in 0.2 mg/mL ascorbic acid in 0.9 % sterile saline, Sigma-Aldrich, Austria) [32, 33]. Only total turns (360°) to the left and to the right were counted. Amphetamine tests were analyzed based on net ipsilateral (left–right) turns and apomorphine tests were analyzed based on net contralateral (right–left) turns [31].

### Tissue processing

After the behavioral recordings were completed, animals were transcardially perfused under deep thiopental anesthesia with phosphate buffered saline (PBS) followed by ice-cold 4 % paraformaldehyde (PFA) (pH 7.4) (Sigma-Aldrich, Austria). Brains were removed and post-fixed in 4 % PFA overnight at 4 °C and then cryoprotected in 30 % sucrose. Subsequently, brains were slowly frozen in 2-methylbutan and preserved at −80 °C until processing. Tissue was sliced on a freezing microtome (Leica, Nussloch, Germany) into 8 coronal series throughout striatal levels (Bregma levels from +1.78 to −2.3).

### Immunohistochemistry

The following antibodies were used in this study: mouse anti-dopamine- and cAMP-regulated phosphoprotein (DARPP-32, 1:5000, BD Biosciences, USA), monoclonal rat anti-CD11b (1:150, Serotec, UK), mouse anti-glial fibrillary acidic protein (GFAP, 1:1000, Millipore, USA), rat polyclonal antibody to human α-syn (15G7, 1:200, Enzo Life Sciences, Germany) and rabbit monoclonal [1536Y] antibody to phosphorylated α-syn (pSyn, 1:1000, Abcam, UK). Secondary antibodies were biotinylated horse anti-mouse IgG and biotinylated goat anti-rat or anti-rabbit IgG (Vector Laboratories, USA). For the visualization of the immunohistochemical binding sites ABC complex (Vector Laboratories, USA) and 3,3’-diaminobenzidine were used. Sections were mounted on slides and coverslipped with Entellan.

### Image analysis

All quantification analyses were done on a Nikon Eclipse E800 microscope equipped with Nikon camera DXM1200 and Stereo Investigator Software (Micro Bright Field Europe, Germany) by an experimenter who was blinded to the genotype of the animals. The optical fractionator method was used to estimate the number of DARPP-32-immunopositive GABAergic medium-sized spiny neurons in the lesioned and the contralateral non-lesioned striatum. The number of GCI-like α-syn inclusion per mm^2^ in 15G7 and pSyn immunostaining was determined in the lesioned and non-lesioned striatum [23, 34]. To analyze astrogliosis (GFAP) and microglial activation (CD11b), the optical density (OD) of the lesioned and non-lesioned striatum was defined at standard camera settings as previously described [35]. GCI density was quantified In any case the area of the striatum was delineated at the respective bregma level according to the Mouse Brain Atlas [36].

### Statistical analysis

After completion of the blinded image analysis the results were de-coded and appointed to the respective experimental group. All statistical analyses were performed using Graph-Pad Prism 5 (Graphpad Software, San Diego, CA, USA) and the results were presented as the mean ± SEM. Five control mice and eight PLP-α-syn mice with successful intrastriatal needle tract placement and identification were included in the statistical analysis. Unpaired *t* test was used for the comparison of the behavioral performance of the two groups. Two-way ANOVA was used with variables genotype (control vs PLP-α-syn) and side (lesioned vs non-lesioned). A P value <0.05 was considered statistically significant.

## Results

### Oligodendroglial α-syn accumulation does not magnify the deterioration of motor performance induced by unilateral QA striatal lesions

Drug-induced rotation behavior resulting from a QA lesion in the left striatum revealed no significant differences between PLP-α-syn and control mice. The number of amphetamine-induced net ipsilateral rotations over a period of 60 min was comparable in PLP-α-syn and control mice (Fig. 1a). As previously reported [31] and expected negligible rotation behavior was induced by apomorphine after a unilateral QA striatal lesion, with no significant difference between PLP-α-syn and control mice (Fig. 1b). General locomotor activity in the vertical (rearing) and horizontal plane in an open field arena showed no differences between QA lesioned PLP-α-syn mice and control mice (*p* > 0.05) (Fig. 1c, d).

**Fig. 1:** Behavioral analysis 15 weeks after unilateral QA lesion in the striatum in PLP-α-syn and control mice. Amphetamine- and apomorphine-induced rotations were presented as net ipsilateral or contralateral turns in a test period of 60 min (**a**, **b**). Open field activity—horizontal and vertical (rearing) were automatically detected over a period of 15 min (**c**, **d**). Data are mean ± SEM

### Oligodendroglial α-syn accumulation does not enhance striatal excitotoxic lesions by focal QA injection

The loss of GABAergic medium-sized spiny neurons induced by 90 nmol QA injections into the left striatum was comparable in PLP-α-syn and control mice (striatal neuronal loss of 247464 ± 54192.97 in QA-lesioned control animals compared to 252596 ± 48682.83 in QA-lesioned transgenic PLP-α-syn MSA animals, Fig. 2).

**Fig. 2:** DARPP-32 neuronal loss in the left striatum after 90 nmol QA injection in PLP-α-syn and control mice. Overview of the unilaterally QA lesioned striatum in control (**a**) and PLP-α-syn mice (**b**) is demonstrated in representative sections at low magnification. In the non-lesioned side immunopositive neurons were easily detectable (*arrows*) at high magnification both in control (**c**) and PLP-α-syn mice (**d**). There was loss of DARPP-32 neurons, identifying only few preserved ones (*arrow*) or some degenerating cell profiles (*arrowheads*) on the lesioned side in controls (**e**) and PLP-α-syn mice (**f**). Statistical analysis with two-way ANOVA showed comparable neurodegeneration in control and PLP-α-syn mice (**g**). Data are presented as mean ± SEM. ***p < 0.001. *L* lesioned side, *NL* non-lesioned side

Excitotoxic insult by QA classically leads to neuroinflammatory response with activation of astroglia and microglia in the lesioned striatum [37, 38]. To assess the glial responses as a measure of the QA lesion extent we measured the optical density of GFAP and CD11b immunohistochemical stainings in the lesioned and non-lesioned striatum, respectively. Astroglial activation was induced by QA in both PLP-α-syn (OD_GFAP_ 0.172 ± 0.012) and control mice (OD_GFAP_ 0.194 ± 0.01) regarding the lesioned striatum with no significant differences in the OD of GFAP immunoreactivity in the striatum between the groups. Regarding the non-lesioned striatum no significant differences between the groups were detected (control mice OD_GFAP_ 0.109 ± 0.004, PLP-α-syn OD_GFAP_ 0.102 ± 0.005) (Fig. 3).

**Fig. 3:** GFAP immunohistochemistry to study astroglial activation due to QA striatal lesion. In the non-lesioned side GFAP-immunopositive astroglial cells were few in number, not activated and easily detectable at high magnification both in control (**a**) and PLP-α-syn mice (**b**). There was intense astroglia activation following QA injection on the lesioned side in both controls (**c**) and PLP-α-syn mice (**d**). Statistical analysis with two-way ANOVA showed comparable astroglial activation in control and PLP-α-syn mice as measured by GFAP optical density (**e**). Data are presented as mean ± SEM. ***p < 0.001. *OD* optical density

Microglial activation tended to be higher in the non-lesioned striatum of PLP-α-syn mice (OD_CD11b_ 0.1 ± 0.014) as compared to control animals (OD_CD11b_ 0.074 ± 0.01), however this difference as measured by the OD of CD11b immunoreactivity in the striatum did not reach significance (Fig. 4). The microglial activation increased significantly in the QA lesioned striatum of both control (OD_CD11b_ 0.166 ± 0.018) and PLP-α-syn mice (OD_CD11b_ 0.191 ± 0.022). Although there was a slight trend towards greater microglial activation in the lesioned striatum of PLP-α-syn as compared to control mice, the difference did not reach statistical significance in terms of OD_CD11b_.

**Fig. 4:** CD11b immunohistochemistry to study microglial activation after QA striatal lesion. In the non-lesioned side CD11b-immunopositive cells were easily detectable at high magnification both in control (**a**) and PLP-α-syn mice (**b**). There was intense microglia activation following QA injection on the lesioned side in both controls (**c**) and PLP-α-syn mice (**d**). Statistical analysis with two-way ANOVA showed comparable intensity of microglial activation in control and PLP-α-syn mice as measured by CD11b optical density (**e**). Data are presented as mean ± SEM. ***p < 0.001. *OD* optical density

Due to the overexpression of human α-syn under the PLP promotor in the PLP-α-syn mice accumulation of α-syn is present in oligodendrocytes (Fig. 5). GCI density was analyzed in non-lesioned (Fig. 5a, b) and lesioned (Fig. 5c, d) striatum of PLP-α-syn mice revealing no statistical significant difference regarding the number of GCIs per mm^2^ (Fig. 5e, f).

**Fig. 5:** GCI-like pathology in PLP-α-syn mice. 15G7 and pSyn immunohistochemistry was applied to visualize GCIs in the non-lesioned (**a**, **b**) and lesioned (**c**, **d**) striatum. Statistical analysis using student’s t test showed comparable density of α-syn-positive GCI-like inclusions in the non-lesioned and lesioned striatum of PLP-α-syn mice with both 15G7 antibody (**e**) and pSyn antibody (**f**). Data are presented as mean ± SEM

## Discussion

Given that not much is known about the etiopathogenesis of MSA and that there is lack of adequate treatment to stop the progression of the disease [1], the understanding of MSA pathophysiology is of tremendous importance. Different approaches have been used in the past aiming to generate MSA mouse models that replicate not only the pathology but also provide insights into the pathogenic mechanisms relevant to the disease [12, 21, 23]. Several studies suggested a role of excitotoxicity in neurodegenerative diseases including MSA [10, 24, 25, 39]. However, it is currently unclear, if pathological aggregation of α-syn in oligodendrocytes may enhance the susceptibility to excitotoxic stress in MSA as it has been shown to be the case with oxidative stress and proteasome dysfunction [12, 23].

The current study, for the first time, characterized the effect of unilateral stereotactic injection of the excitotoxin QA into the striatum of the transgenic PLP-α-syn mouse model of MSA to assess whether excitotoxic insult may be aggravated by oligodendroglial α-syn pathology. The excitotoxic lesion of the striatum of transgenic PLP-α-syn mice was comparable to the one induced by the same treatment paradigm in control mice as measured by functional and neuropathological readouts. Therefore, it can be concluded that the occurrence of α-syn aggregates in oligodendroglial cells in the transgenic PLP-α-syn mouse does not potentiate the effect of QA excitotoxicity on medium-sized spiny striatal neurons compared to control mice at 7 months of age.

Although a tendency toward lower number of GABAergic medium-sized spiny neurons was seen in the non-lesioned striatum of PLP-α-syn mice versus controls, the difference was not significant. The additional excitotoxic insult induced by intrastriatal injection of 90 nmol QA did not reveal differences in the vulnerability of striatal neurons to NMDA mediated toxicity in the presence or absence of oligodendroglial α-syn pathology. In both cases (transgenic and non-transgenic mice) striatal neuronal loss was about 70 %. It is interesting to note that in contrast to QA, another classically selective striatal neurotoxin with a different mode of action, i.e. 3-NP systemically applied—a mitochondrial complex II inhibitor—, shows increased striatal toxicity in PLP-α-syn mice and furthermore induces neuronal loss in regions (cerebellum, pons, inferior olives) that are classically not affected by 3-NP toxicity in wild type mice [12]. These differences in the vulnerability to QA and 3-NP of PLP-α-syn mice may reflect the divergent actions of the two neurotoxins. It is possible that the wide-spread mitochondrial dysfunction linked to systemically applied 3-NP treatment may influence the oligodendroglial support of neurons, which leads to neuronal loss in additional brain regions. In contrast, QA appears to trigger primary striatal neuronal death through NMDA mediated excitotoxicity without significant contribution of the oligodendroglial α-synucleinopathy in this context. This notion is supported by the finding that QA lesion did not significantly affect the density of GCIs in the striatum. We cannot exclude, however, that the different mode of application of the toxins (sub-chronic systemic for 3-NP versus acute local intracerebral for QA) may also contribute to the observed responses. Furthermore, we cannot exclude that intracerebral QA injections of 90 nmol into the striatum might have been too severe and therefore masked a further potentiation of the lesion size by the oligodendroglial α-syn pathology in the PLP-α-syn mouse model. In addition, at this stage it cannot be excluded that the age of the transgenic animals might interfere with the vulnerability to QA.

The similar unilateral striatal lesion size in PLP-α-syn and control mice was consistent with the behavioral readouts. Similar to previous reports [31] the QA unilateral striatal lesion in both control and PLP-α-syn mice induced comparable modest ipsilateral turning under amphetamine and no net rotational bias under apomorphine treatment. Classically doses lower than 0.5 mg/kg b.w. apomorphine can efficiently induce contralateral rotations in the unilateral 6-OHDA mouse model, where hypersensitivity of the dopamine receptors in the unilateral striatum is present [40]. However, in the QA lesion model apomorphine is expected to induce ipsilateral rotations due to the activation of striatal dopamine receptors in the non-lesioned side. We cannot exclude that higher drug doses might have been able to trigger apomorphine-induced rotations in the current QA lesion paradigm. Although the rotational data were normally distributed in the present study, we observed high intragroup variability of the rotation behavior that may reflect some variability in the precise location of the neostriatal lesion as suggested in earlier studies [31]. Previous reports in the QA model of HD [41] have suggested effects of the unilateral excitotoxic lesion on the rearing open field behavior. The current results demonstrate that α-syn oligodendroglial pathology does not have a cumulative effect with the QA insult in the transgenic MSA model to affect either rearing or horizontal activity in an open field arena.

An important feature of the excitotoxic lesions induced by QA is the neuroinflammatory response usually estimated by astroglial and microglial activation [37, 38]. We observed a similar degree of astroglial activation as measured by GFAP immunoreactivity optical density in PLP-α-syn and control mice due to the unilateral QA striatal lesion. Consistent with our previous work microglial activation assessed by optical density of CD11b immunoreactivity tended to be increased in the non-lesioned striatum of transgenic versus control mice but QA lesion was not associated with a significant difference in the microglial response between PLP-α-syn and control mice supporting the notion of lack of a significant cumulative effect between oligodendroglial α-syn accumulation and excitotoxic insults.

In the PLP-α-syn mouse model α-syn is expressed under the oligodendroglial promoter PLP and mice feature GCI-like inclusion pathology as shown previously [12, 42]. Furthermore, pathological α-syn accumulation is already present in the PLP-α-syn mouse model at the age of 7 months as shown here. In the current study, we did not observe changes in the accumulation of α-syn in the PLP-α-syn model upon striatal stereotaxic injections of QA suggesting that QA does not influence α-syn aggregation pathology in oligodendroglial cells. This finding further implies the absence of significant cumulative effects between an excitotoxic insult and oligodendroglial α-syn accumulation.

## Conclusions

In conclusion, here we report for the first time the impact of a striatal excitotoxic insult in the PLP-α-syn mouse model of MSA. Taken together, the present data suggest that QA induces severe striatal neurodegeneration without any difference between transgenic and control mice. Therefore, the current results do not support a cumulative effect of oligodendroglial α-syn accumulation and excitotoxicity to induce MSA-like neurodegeneration in contrast to oxidative or proteolytic stress [12, 23].
